RETRACTED

# Comparison of Outcomes of Percutaneous Nephrolithotomy (PCNL) Between Adults and Pediatrics Population: A Single-Center Retrospective Study

**DOI:** 10.7759/cureus.22690

**Published:** 2022-02-28

**Authors:** Muhammad Rizwan Umer, Marina Basta, Sandrine Kakieu Djossi, Amin Tafti, Musharaf Khan, Maria Binte Sarfraz, Sabeen Sharif Khan, Jobby John, Khizer Shamim

**Affiliations:** 1 Medical School, District Head Quarter Hospital, Nankana Sahib, PAK; 2 Medical School, St. George's University, True Blue, GRD; 3 Medical School, California Institute of Behavioral Neurosciences and Psychology, Fairfield, USA; 4 Medical School, Virginia Commonwealth University, Richmond, USA; 5 Neurosurgery, Combined Military Hospital, Rawalpindi, PAK; 6 Physiology, Army Medical College, National University of Medical Sciences, Rawalpindi, PAK; 7 Medicine, Aga Khan University Hospital, Karachi, PAK; 8 Internal Medicine, Dr. Somervell Memorial CSI Medical College, Thiruvananthapuram, IND; 9 Medical School, Ziauddin University Hospital, Karachi, PAK

**Keywords:** comparison, sfr, adults, children, pcnl

## Abstract

Introduction: Percutaneous nephrolithotomy (PCNL) has almost completely replaced open surgery for kidney stones because of continuous advancements in the method since the first PCNL was performed in 1976. The aim of this study is to compare the characteristics and outcomes of adult patients and pediatric patients who had undergone PCNL.

Methodology: A retrospective study was conducted at the Sindh Institute of Urology and Transplantation (SIUT) Hospital in Karachi, Pakistan. It included the data of patients who underwent PCNL from January 2015 to January 2022 at the SIUT hospital. The primary outcome variable was the stone-free rate (SFR). Secondary outcomes included length of hospital stay, and complications were assessed using modified Clavien classification system

Results: There is no significant difference in the SFR at discharge between pediatric and adult patients (86.67% vs 88.69%, p=0.634). There is no significant difference between the two groups in relation to the total length of hospital stay (p=0.446). Moreover, 12.50% and 11.11% of adults and children developed complications, respectively, after the procedure. The percentages are not significantly different between the two groups (p=0.266).

Conclusion: The current study using standardized and consistent PCNL techniques shows that SFR is similar in both adults and children, and there is no difference in complications between adults and children.

## Introduction

Percutaneous nephrolithotomy (PCNL) has almost completely replaced open surgery for kidney stones because of continuous advancements in the method since the first PCNL was performed in 1976 [1]. Despite the advantages of PCNL over open surgery, the rates of complication for this procedure remain high [2].

RETRACTED

Moreover, because of the higher incidence of anatomical and metabolic abnormalities in pediatric stone patients, residual stones after extracorporeal shock wave lithotripsy (ESWL) can cause recurrence [3]. The other major concern in children is avoiding the retreatment need. As a result, all treatment choices for achieving stone-free status in this age group are critical and should not be limited or excluded [4]. Therefore, the ideal treatment needs to be minimally invasive with a lower retreatment rate and high stone clearance.

Several studies have shown that PCNL is effective and safe in children, but most of these studies are limited to case series, and several studies did not have a control group for comparison [5,6]. Several surgical principles incorporated in PCNL were developed in adults, but these principles directly applied to children [7]. One of the critical considerations is the smaller size of the urinary tract. Children have taken to techniques that use narrower access tracts, such as mini-perc, ultra-mini perc, and micro-perc [8,9]. The reduced blood volume and increased risk of hypothermia from irrigation solutions are other technical problems peculiar to children undergoing PCNL [10]. Furthermore, differences in outcomes after renal stone surgery between adults and children can also exist. According to the study conducted by Zeng et al., children had a greater stone-free rate (SFR), needed fewer access tracts, and had a shorter nephrostomy tract [7].

PCNL is only conducted at a few specialized centers in Pakistan's main cities. Due to technical challenges and fear of consequences and procedure failure, there is substantially higher apprehension among the pediatric population. In the current research, we aimed to compare characteristics and outcomes of adult patients and pediatric patients who had undergone PCNL.

## Materials and methods

A retrospective study was conducted at the Sindh Institute of Urology and Transplantation (SIUT) hospital in Karachi, Pakistan. It included the data of patients who underwent PCNL from January 2015 to January 2022 at the SIUT hospital. Patients were divided into two groups based on World Health Organization (WHO) age classification criteria. Two groups included pediatrics, zero to 14 years old, and adults, more than 14 years old [7]. Clinical data, including the age of patients, gender, stone size, comorbidities, operation time, side of surgery, and number of stones, were extracted from the hospital management information system (HMIS). The time between the first renal puncture and the completion of the stone removal was considered the operation time.

RETRACTED

All procedures were done under general anesthesia by surgeons. Under fluoroscopic supervision, an open-end catheter was passed cystoscopically up to the renal pelvis in a lithotomy position. After that, the patient was placed in a prone position. Under fluoroscopic supervision, the pelvicalyceal system was pierced with a 23 Fr spinal needle. The gliding wire was inserted into the pelvicalyceal system through a spinal needle. Metallic dilators were used to dilate the tract over gliding wire. Under fluoroscopic guidance, a 30 Fr PCNL sheath was inserted into the pelvicalyceal system over metallic dilators. The PCNL sheath was then used to introduce a 26 Fr nephroscope. Standard procedures were used in both children and adults. The stones were broken with a pneumatic lithoclast, and the stone fragments were extracted with a three-prong grasper. All patients had their nephrostomy tubes sized 4 to 6 Fr; the tubes were passed and withdrawn on the second postoperative day.

The primary outcome variable included the stone-free rate (SFR). SFR was defined as no residual stones 3 mm on postoperative kidney ureter bladder (KUB) radiography, nephrostogram, ultrasound, or computed tomography (CT). SFR is categorized into two groups (yes and no) based on the above-mentioned definition of SFR. Secondary outcomes included length of hospital stay, and complications were assessed using a modified Clavien classification system [11].

Statistical analysis

Data analysis was done using STATA version 16.0 (College Station, TX: StataCorp LLC). Student's t-test was used to compare continuous variables in two groups, while chi-square test was used to compare proportion between two groups. P-value <0.05 was considered statistically significant.

## Results

Two hundred fifty-eight patients entered the study. A total of 168 (65.15%) patients were adults and 90 (34.88%) were children. Table 1 shows the characteristics of patients. The majority of patients were males in both adults (69.64%) and children (76.67%). The mean stone size was 38.03 ± 18.91 mm in adults and 23.74 ± 14.33 in children (p=0.001). Regarding complications, adult patients had higher comorbidities as compared to the pediatrics group (p=0.001). In addition, 33.93% of patients in the adult group had previous stone-related surgery compared to 27.78% of patients in the children group (p=0.312). The operative time was significantly higher in the adult group (85.44 ± 27.83 minutes) than in the children group (68.50 ± 28.68 minutes) (p=0.001). There is no significant difference between the two groups in relation to the side of surgery (p=0.108).

RETRACTED

**Table 1:** Comparison of characteristics between adults and paeds. *Mean (standard deviation). **P-value significant at <0.05.

Variables						Adults n (%)	Paeds n (%)	p-Value
Age*						35.75 ± 15.30	7.76 ± 3.66	0.001**
Gender					Male	117 (69.64)	69 (76.67)	0.213
					Female	51 (30.36)	21 (23.33)	
Side of surgery				Left		72 (42.86)	48 (53.33)	0.108
				Right		96 (57.14)	42 (46.67)	
Stone size (mm)*						38.03 ± 18.91	23.74 ± 14.33	0.001**
Comorbidities			No			114 (67.89)	88 (97.78)	0.001**
			Yes			54 (32.14)	2 (2.22)	
Previous stone-related surgery		No				111 (66.07)	65 (72.22)	0.312
		Yes				57 (33.93)	25 (27.78)	
Duration of surgery (minutes)*						85.44 ± 27.83	68.50 ± 28.68	0.001**
Number of stones	1					118 (70.24)	64 (71.11)	0.883
	>1					50 (29.76)	26 (28.89)	

Regarding study outcomes, there is no significant difference in the SFR at discharge between pediatric and adult patients (86.67% vs 88.69%, p=0.634). There is no significant difference between the two groups in relation to the total length of hospital stay (p=0.446). Moreover, 12.50% and 11.11% of adults and children developed complications, respectively, after the procedure. The percentages are not significantly different between the two groups (p=0.266). Ten complications were reported in children. Common complications among children included fever (n=4), vomiting (n=3), postoperative pain (n=2), and blood transfusion (n=1). On the other hand, 21 patients in the adult group reported complications. Most common grade 1 complications were fever (n=6), vomiting (n=5), and postoperative pain (n=8). Grade 2 complication included blood transfusion (n=2). Modified Clavien classification system has five categories of complications. Grade 1 represents minor while grade 5 represents critical; grades 3a and 3b are part of this classification system. Table 2 shows the comparison of outcomes between pediatric and adult groups.

**Table 2:** Comparison of outcomes between adults and paeds. *Mean (standard deviation). SFR: stone-free rate

Variables		Adults n (%)	Paeds n (%)	p-Value
SFR	No	149 (88.69)	78 (86.67)	0.634
	Yes	19 (11.31)	12 (13.33)	
Length of stay (days)*		4.25 ± 5.08	4.67 ± 5.08	0.446
Complications				
All		21 (12.50)	10 (11.11)	0.266
Grade 1		19 (11.30)	9 (10.00)	0.544
Grade 2		2 (1.90)	1 (1.11)	0.699
Grade 3a		0 (0)	0 (0)	
Grade 3b		0 (0)	0 (0)	
Grade 4		0 (0)	0 (0)	
Grade 5		0 (0)	0 (0)	

## Discussion

The treatment of kidney stones in children is evolving. Any kind of treatment demands balances between the complications associated with the procedure and SFR. ESWL has been used to treat stones in the upper urinary system that are less than 20 mm in diameter. Stones greater than 20 mm were also managed using ESWL in children, but only 50% of children were stone free at discharge with ESWL [12]. In children with large upper urinary tract stones, PCNL is an effective therapy of choice. The less robust and smaller pelvicalyceal system, renal hypermobility, and children's lesser tolerance for blood loss were some of the characteristics that made this treatment more difficult.

RETRACTED

A study conducted by Badawy et al. found that SFR in children after a single treatment session is 83.3% [13]. Another study included 135 children conducted by Salah et al. reported an SFR of 98.5%, and complications included 0.7% of blood transfusion and 8% urine leakage [14]. All these studies did not have any comparison group. Considering the differences in the size of the urinary tract between adult and pediatric patients, our study has determined whether this would create an impact on the efficacy of PCNL among children. Our study did not find any significant difference in SFR at discharge between adult and pediatric patients. In addition, the current study did not find any significant difference in length of stay between adult and pediatric patients undergoing PCNL. The study conducted by Zeng et al. also found similar results [7]. Even though several studies have not compared the outcomes of PCNL between pediatrics and adult patients, it has been found that SFR in the pediatrics group ranges up to 100% [15,16].

One of the important issues in any PCNL included complications, especially in children. In our study, grade 2 complications in children were reported in 1.11% compared to 1.90% in adults, and there is no significant difference between the two groups. The study conducted by Zeren et al. reported a 24% blood transfusion rate, 30% postoperative fever, and 87% SFR in children undergone PCNL, but the study did not contain any comparison group [17]. Our study is the first one in Pakistan to utilize the Clavien system for comparison of complications of PCNL in adults and children. As per the Clavien classification, complications were reported in 30% of children by Ozden et al. [18] and 29.2% of adults by Tefekli [11]. Our study found that overall complications in children and adults were 12.50% and 11.11%, respectively. Besides this, there were no high-grade complications in any of the two groups.

In our study, no difference was there in the longevity of hospital stay between the two groups. Similar findings were also reported in the study conducted by Iqbal et al. [19]. In addition, the mean operative time in children is shorter than in adults. Because operating time is experience-dependent and depends on the competence level of surgeons and the number of surgeries performed at a given center, operative time varies among studies [20].

RETRACTED

Considering the efficacy and safety of PCNL in children, it should be a standard of care in adults and children for the management of kidney stones. Technical difficulties and lack of experience need to be overcome as the current study ruled out any difference with respect to outcome, operative difficulties, and postoperative complications.

The current study has certain limitations. First, our data came from a single high-volume center, and it's possible that it's not applicable to all. Furthermore, there is a scarcity of long-term data on PCNL's impact on stone recurrence. Future research should use a prospective design with longitudinal follow-up from various centers.

## Conclusions

The role of PCNL is very important in the management of pediatrics and adult patients with a large burden of kidney stones. PCNL's technical ideas that have been successfully applied to children were developed in adults. The current study using standardized and consistent PCNL techniques shows that SFR is similar in both adults and children, and there is no difference in complications between adults and children. It shows that PCNL is a safe and effective procedure in the management and treatment of large stones among children.
